# International trade and finance exploration using network model of computer trade platform

**DOI:** 10.1371/journal.pone.0260883

**Published:** 2021-12-03

**Authors:** Yi Zhang, Yi Yuan

**Affiliations:** 1 School of Management, XI’AN University of Finance and Economics, Xi’an, Shaanxi, China; 2 School of Business, XI’AN University of Finance and Economics, Xi’an, Shaanxi, China; Ministry of Natural Resources North Sea Bureau, CHINA

## Abstract

International trade becomes increasingly frequent with the deepening of economic globalization. In order to ensure the stable and rapid development of international trade and finance, it is particularly crucial to predict the sales trend of foreign trade goods in advance through the network model of computer trade platform. To optimize the accuracy of sales forecasts for foreign trade goods, under the background of "Internet plus foreign trade", the controllable relevance big data mining of foreign trade goods sales, personalized prediction mechanism, intelligent prediction algorithm, improved distributed quantitative and centralized qualitative calculation are taken as the premise to design dynamic prediction model on export sales based on controllable relevance big data of cross border e-commerce (DPMES). Moreover, after the related experiments and comparative discussions, the forecast error ratios from the first quarter to the fourth quarter are 2.3%, 2.1%, 2.4% and 2.4% respectively, which are also within the acceptable range. The experimental results show that the design combines the advantages of openness and extensibility of Internet plus with dynamic prediction of big data, and achieves the wisdom, quantitative and qualitative prediction of the volume of goods sold under the background of "Internet plus foreign trade", which is controlled by the relevant data of foreign trade. The overall performance of this design is stronger than the previous models, has better dynamic evolution and high practical significance, and is of great significance in the development of international trade and finance.

## Introduction

Under the background of world economic globalization, international trade is of great significance for a country to increase its foreign exchange reserves and enhance the market space and market competitiveness of its enterprises. Meanwhile, it provides massive resources to meet the domestic needs, which can accelerate the development of capital circulation in the financial field, and then feed back to the good development of international trade, so as to form a good cycle and promote the development of international trade and finance. In international trade, the structure of foreign trade under the background of "Internet plus foreign trade" is not single. The future form of goods is subject to supply and demand and various conditions. "Internet plus foreign trade" has the advantage of forecasting information., and it can easily predict the sales volume of foreign trade goods. Therefore, the network model of computer trade platforms currently has become the focus of multiple fields.

Niu et al. (2021) [1] used some big data classification methods to collect a large amount of foreign trade information and analyze the future trend of commodity supply and demand. There is also the establishment of goods sales analysis model through the previous information of foreign trade, and the correlation analysis model proposed by using quantitative and qualitative analysis methods according to historical information and other relevant points.

The above research has some reference significance, because the word "Internet plus" does not appear for a very long, and it is not well realized. The advantages of online information prediction of Internet plus are not revealed. Moreover, how to make use of big data in the prediction of the dynamic intelligence of foreign trade goods sales in the context of "Internet plus foreign trade" has not yet been relatively well studied. According to the current research status, computer trade platform is taken as the premise. Then, from the aspect of controllable relevance big data mining of foreign trade goods sales under the background of "Internet plus foreign trade", a quantifiable, dynamic and intelligent dynamic prediction model on export sales based on controllable relevance big data of cross border e-commerce (DPMES), driven by the Internet plus foreign trade, is constructed. The purpose is to achieve the dynamic prediction target of export sales volume, which can guide foreign trade enterprises in marketing and optimizing inventory strategy, and also promote the development and research of Internet plus, big data and foreign trade technology, so as to provide the basis for maintaining the high-speed and stable development of international trade and finance.

## Materials and methods

### Overall framework of computer trade platform network model

#### Controllable relevance big data mining of foreign trade goods sales

Controllable relevance refers to the controllable and interrelated nature of multiple elements that affect the research data. Under the background of "Internet plus foreign trade", based on the export-related data, the big data mining must first be based on the Internet plus foreign trade background platform to excavate the data such as policy, goods category and so on. Fig 1 displays the details.

**Fig 1:** Big data mining content.

It is essential to mine the core points and controllable relevance big data that play a relevant role in the sales volume prediction of export goods. Figs 2–4 are its model.

**Fig 2:** Business operation module of controllable relevance big data mining model of foreign trade goods sales under the background of "Internet plus foreign trade".

**Fig 3:** Technology environment module of controllable relevance big data mining model of foreign trade goods sales under the background of "Internet plus foreign trade".

**Fig 4:** Mining process module of controllable relevance big data mining model of foreign trade goods sales under the background of "Internet plus foreign trade".

The model consists of three parts. The detailed mining process and method are as follows:

The first step is to build the premise of prediction behavior, dynamic classification and estimation function of big data.

The controllable relevance index information acting on prediction is predicted and divided, and the goal of information mining is clarified. Previous scholars have practiced the relevant methods of big data classification, but they have not clearly described the fuzzy phenomenon of data and combined with internet thinking [2], which has no ability of dynamic classification of Internet big data. Here, it is particularly essential to improve and upgrade. The information dynamic classification and prediction scheme based on prediction behavior are described [3].

Assumption: It is known that the scope C of data mining theory and its non-empty subset *A*, (*C*, *A*) = {(*C*_*i*_, *A*_*i*_)|*i*∈*N*_+_} refer to the set of credibility measures; *S* = {*S*_*i*_ = (*S*_*i*1_, *S*_*i*2_, *S*_*i*3_)|*i*∈*N*_+_} refers to the total data of other platforms on the Internet plus foreign trade, including n elements. *SAM* = {*SAM*_*i*_|*i*∈*N*_+_} and *SAB* = {*SAB*_*i*_|*i*∈*N*_+_} are the set of data fuzziness and uncertainty respectively; the mapping function of classification subject and object is:*F*1 = (*FS*_*i*_→*FC*_*i*_). If, $\exists C_{i}\in C\wedge (C_{i},\;A_{i})\wedge (S_{i1},\;S_{i2},\;S_{i3})\wedge SAM\wedge SAB\neq False$, the function in Eq (1) can be used as the premise of the dynamic classification and estimation method of information predicting behavior. CF(i) is recorded as:

$$CF(i)=\frac{(1,\;n)\cdot |S_{i}|\cdot |FSi|\cdot I_{uv}\mu (vi)\cdot \sum_{i=1}^{n}SAM_{i}}{(I_{uv},\;I_{u},\;I_{v})\cdot \mu (u_{i})\cdot |C_{i}|\cdot |FC_{i}|\cdot |A_{i}|\cdot \sum_{i=1}^{n}SAB_{i}}$$ (1)

The improved CF (i) maps the fuzzy phenomenon and uncertainty phenomenon to the corresponding (C_i_, A_i_) respectively. Unlike previous methods, this method can better explain the fuzziness and uncertainty of dynamic classification of Internet big data.

The second is to build the association rule function, find out the internal association regularity of controllable relevance big data [4], and then sort out the available data sources. In the past, some people have proposed relevance grouping rules, but the proposed rules only have simple relevance to the data, and the relevance is not high enough. Hence, it is essential to improve it and establish a more accurate association rule function [5].

On the premise of Eq (1), it is assumed that K1 and K2 are possibility space and necessity measure space respectively [6]; the constraint time of S_i_ in A is t_i_, and *ξ* is recorded as the fuzzy variable in K1 [7]; at this moment, the correlation expectation E (x) between the correlation degree J_i_ and the uncertainty variable x is b [8], and the threshold is ω_0_. The constraint time conforming to the mapping " *G*:*K*1+*K*2→*K*1∙*K*2" represents the optimal search time T_i_; the correlation error is recorded as Eq (2):

$$e(S_{i,}S_{j})=b-\sum_{x=i}^{j}E(x)$$ (2)

Eq (3) is a perfect association rule.


$$C{V(S}_{i,}S_{j})=\frac{\sum_{i=1}^{n}\sum_{j=1}^{m}e(S_{i},S_{i})\cdot \xi \cdot (|CFi(i)-K1|)}{w_{0}\cdot \prod_{i=1}^{n}(K2\cdot t_{i}T_{i}\cdot J_{i})}$$ (3)

The function of the improved Eq (3) is reflected in the internal correlation regularity of controllable correlation big data of export goods sales.

The third step is to construct online k-means clustering and description functions with better clustering ability [9], so that the similarity of classified controllable correlation big data becomes higher. In previous online clustering schemes, the classified data blocks obviously have cross-border behavior [10]. K-means clustering scheme has the ability of association clustering. Therefore, the following will learn from these two methods to improve and propose an online K-means clustering and description scheme.

Under the premise of Eq (3), the weight of a prediction subject and object recommendation is set as ω_1_ and ω_2_; the cluster recommendation set is TJ = {tj_1_, tj_2_, …, tjn}, the associated expected value is Qx (tj_i_, tj_j_) = TS (SAM_ii_, SAB_i_)·e(S_i_, S_j_), entropy is Qn (tj_i_, tj_j_) = TS (SAM_ii_, SAB_i_) +e (S_i_, S_j_), and super entropy is Qe (tj_i_, tj_j_) = TS (SAM_ii_, SAB_i_) /e (S_i_, S_j_). Then, Eq (3) displays the improved online k-means clustering and description method:

$$CVV(S_{i},S_{j})=\frac{Qx(tj_{i},\;tj_{j})\cdot \sum_{i=1}^{m}\sum_{j=1}^{n}\cdot (tj_{i}\cdot tj_{j}\cdot |\omega_{i}\cdot TJ|)}{Qn(tj_{i},\;tj_{j})\cdot Qe(tj_{i},\;tj_{j})\cdot CV(S_{i},\;S_{j})}$$ (4)

The improved Eq (4) can effectively classify the sale data block of similar cross-border trade goods of "Internet plus foreign trade".

The fourth is to learn from some characteristics of the previous network information matching principles [11, 12] to achieve the integration of key factors, so as to solve the disadvantages of inter-domain mapping [13].

#### Personalized prediction mechanism

The model in Fig 1 is adopted to form the following prediction scheme:

"Incremental evolution—integration" prediction mechanism. The neural network method is adopted to realize the incremental dynamic evolution and integrate good prediction. Here, the incremental evolution factor attribute can be recorded as (B_n_)^2^ tuple Q = (mathematical combination of B_n-1_ and B_n_), and the combination number M1 = ω_i_CE(R_n_)^2^. “Random distribution–correlation” prediction mechanism. Machine learning is used to correlate the randomly distributed big data of goods sales and then predict [14]. Here, the random distribution factor attribute can be recorded as (B_n_)^2^ tuple Q = (mathematical combination of B_n-1_ and B_n_), and the combination number M_2_ = CE`(R_n_)^2^. In order to realize personalized estimation quantitatively and qualitatively, these two mechanisms should be expressed in mathematical form. C&M-CVPDSS (Case-based and Multiplicative analytic hierarchy process-based Customer Value Prediction Decision Support System) well expresses this mechanism.

Eqs (5) and (6) display the mathematical functions of "Incremental evolution—integration" prediction mechanism and “Random distribution–correlation” prediction mechanism.


$$DT=\frac{\sum_{i=1}^{n}\sum_{j=1}^{m}\left(|CER(C_{i}C_{j})|\cdot |B_{j}|/G(C_{i},\;C_{j})\right)}{Q\cdot B_{n}^{2}\cdot AA\cdot CVV(S_{i},S_{j})}$$ (5)

$$DTT=\frac{\sum_{i=1}^{n}\sum_{j=1}^{m}\left|A_{i}\cdot CVV(S_{i},\;S_{j})\cdot G(C_{i},\;C_{j})|/B_{j}\right)}{DT\cdot Q\cdot B_{n}^{2}\cdot CER(C_{i}C_{j})}$$ (6)

Among them, DT is the mechanism to automatically realize the transformation from complex incremental evolution and integration indexes to relevant details; DTT is a mode transformation from abstract random distribution, association index and similarity evaluation to relevant details. Eqs (5) and (6) automatically realize the transformation from an abstract random distribution, association, evolution, integration index and similarity evaluation to specific mechanism and mode [15].

#### Intelligent prediction algorithm of DPMES

First, CF (i) is solved according to Eq (3) to predict the target. When the solution of CF (i) is not empty set, the resource planning, design and integration strategy of controllable relevance export goods sales information prediction under the "Internet plus foreign trade" background is expressed as Eq (7):

$$\left(C_{i},\;A_{i}):\;\{(C,\;A)\}\overset{CF(i)}{↔}FS_{i}:\;\{FC_{i}|i\in N_{+}\right\}$$ (7)

The controllable relevance prediction influence elements are obtained through Eq (7), and the dynamic intelligence classification makes the prediction entities have a strict physical mapping relationship [16].

Second, the integration strategy of dynamic prediction intelligence is discussed, and the prediction components are deleted online. The value range of the fuzzy variable is obtained according to Eq (3). Among them, the highest value DT_max_ of DT and the lowest value DTT_min_ of DTT are adopted to find out the prediction components that meet the definition domain of [DTT_min_, DT_max_]. The integration strategy is expressed by the constraint coefficient λ as Eq (8):

$$\lambda =\frac{\left(C_{i},A_{i}\right)}{FS_{i}:FS_{i}}$$ (8)

Third, according to Eq (8), in K1 and K2, any ξ conforming to the threshold ω_0_ in (C, A) is found to obtain the optimal search time T_i_. Eqs (3) ~ (4) are adopted to obtain the controllable correlation and regularity of data. On the premise of the identification of the good failure prediction method, a dynamic prediction and evaluation integration strategy of controllable relevance export goods sales information is proposed [17]. Eq (8) displays its function, which is to calculate the membership M (S_i_, S_j_) of CVV (S_i_, S_j_) for dynamic optimization integration of Qn (tj_i_, tj_j_):

$$M(S_{i},\;S_{j})=CVV(S_{i},\;S_{j})\cdot \lambda \cdot DT\cdot DTT$$ (9)

Fourth, according to the incremental evolution factor attribute and random distribution factor attribute of Eqs (5) ~ (6), the prediction behavior category is BT. The deviation between the target prediction score and the actual score is MAE, and the similarity among clusters is the lowest. When the similarity between μ (x) and μ (y) reaches the highest value, several target prediction behaviors with different scoring characteristics will be attributed to the behavior set with different membership degrees to achieve collaborative filtering recommendations [18].

Fifth, as the core algorithm of the previous algorithms, the distributed quantitative, centralized and qualitative online optimization prediction scheme has been found [19]. In the past, quantitative and qualitative methods are used for online optimization, but they cannot optimally solve the disadvantages of distributed and centralized optimization calculation. The multiple linear regression method adopts a two-dimensional table according to the key factors, which can eliminate the problems of distributed, centralized and correlation prediction of data. Therefore, the following improvements are made to the quantitative and qualitative methods on the premise of this method. All M (S_i_, S_j_) is obtained according to Qe (tj_i_, tj_j_), and all nodes flexibly select the next cluster head node according to the current position of all its neighbor nodes.

In this regard, the clustering, segmentation and isolation points are respectively expressed as Eqs (10)—(12) in turn:

$$HQ=\frac{{\left(\mathrm{CV}\;{\left(S_{i},S_{i}\right)}^{T_{i}}\right)}^{-1/4}{\left(DT^{T_{i}}\right)}^{-1/2}{\left(CF{\left(i\right)}^{T_{i}}\right)}^{-1/3}}{M(S_{i},S_{j})}$$ (10)

$$HF={\left(FS_{i}^{Ti}\right)}^{-1/3}{\left(CVV{\left(S_{i},\;S_{j}\right)}^{Ti}\right)}^{-1/2}{\left(DTT^{T_{i}}\right)}^{-1/4}$$ (11)

$$HG=CVV{\left(S_{i},\;S_{j}\right)}^{\lambda /2}CV{\left(S_{i},\;S_{j}\right)}^{\lambda }{\left(DTT^{\lambda }\right)}^{-1/3}$$ (12)

Hence, the distributed quantitative calculation and centralized qualitative calculation functions are presented in Eqs (13) and (14) in turn, which can quantitatively and qualitatively predict the sales volume of export goods.


$$TCL(S_{i})=\frac{HG\cdot |CF(i)|\cdot \sum_{x=1}^{n}\left(CV(S_{i},\;S_{j})\cdot DTT\right)}{HF\cdot FS_{i}\cdot DT\cdot \prod_{x=1}^{n}\left(\lambda \cdot CVV(S_{i},\;S_{j}\right)}$$ (13)

$$TCX(S_{i})=\frac{HQ\cdot |M(S_{i},\;S_{j})|\cdot FSi\cdot \sum_{x=1}^{n}CV(Si,\;Sj)}{CVV(S_{i},\;S_{j})\cdot DTT\cdot \prod_{x=1}^{n}\left(\lambda \cdot TCL{(S}_{i}\right)}$$ (14)

Sixth, (C_i_C_j_) _max_ and (C_i_C_j_) _min_ represent the highest and lowest values of C_i_C_j_. Steps 1 to 5 are repeated for many times to fix the code feature C_i_C_j_ of C_i_ in the threshold interval [ω_i_, ω_j_]. Whether (*C*_*i*_*C*_*j*_)_*max*_>*ω*_*i*_∧(*C*_*i*_*C*_*j*_)*min*<*ω*_*j*_ holds is determined. If it holds, Eq (10) is adopted to search the normal controllable relevance big data of goods from the huge big data, and establish a distributed quantitative calculation system to obtain quantitative prediction data; If not, Eq (14) is applied to the problem cluster to be solved in time and space to form a centralized qualitative intelligent prediction model.

Seventh, the parallel comprehensive prediction function equation presented in Eq (15) is constructed:

$$TCZ(S_{i})=TCX{\left(S_{i}\right)}^{\lambda }\cdot TCL{\left(S_{i}\right)}^{T_{i}}$$ (15)

At this point, the algorithm is completed.

### Construction of network model of computer trade platform

The previous personalized prediction mechanism and intelligent prediction algorithm are used. A decision tree is adopted to design the DPMES model, as shown in Fig 5.

**Fig 5:** DPMES model.

The design process is shown below:

The first step is to define the prediction direction and select the data range required for modeling according to the first step of the intelligent prediction algorithm, and then screen and obtain the relevant factors with prediction conditions.

The second step is to find the controllable relevance core factor according to steps 2 ~ 3 of the intelligent prediction algorithm, and detect the consistency, controllable relevance and regularity of the core feature number sequence. Then, it is essential to quantify the incremental evolution and integration relationship within the key influencing factors of export goods sales with random distribution. λ is adopted to dynamically delete prediction components. Key factors are integrated and data are processed [20].

The third step is to achieve collaborative filtering recommendation according to algorithm step 4 and classify the subset of prediction behavior.

The fourth step is to dynamically predict the future sales trend of export goods according to Eqs (13) ~ (15) [21].

Finally, the model is evaluated and applied. The error analysis is given to the prediction data of various prediction methods. Fig 5 presents the specific process.

### Experimental data collection

The data used are 10000 sets of relevant data and related information about the export of the manufacturing industry from the platform of the ministry of foreign trade and economic cooperation, including the Internet plus foreign trade platform. According to the controllable relevance big data model of the cross-border export sales under the background of "Internet plus foreign trade", the keywords are analyzed from the direction of "sales attention" and "factor concern". One week is a cycle. Figs 6 and 7 display relevant information.

**Fig 6:** Experimental data analysis of sales attention (A: product category; B: total customer demand; C: customer buying psychology; D: product life; E: in stock; F: price; G: Logistics; H: risk).

**Fig 7:** Analysis of experimental data of factor attention.

Experiment 1 is to use the above 10000 groups of relevant data to prove that the improved scheme has relevant advantages. The process is as follows:

The first is to check that the data information of goods v must be controllably associated with goods u, and to test the validity of Eqs (1) ~ (12).

The second is to test Eqs (13) ~ (15) of distributed quantitative, centralized qualitative prediction and parallel comprehensive prediction function.

The inspection indexes include reconfiguration error (the rematching difference stored in the export goods sales volume big data), feature point error (the difference in the controllable relevance feature matching of export goods sales volume), and mismatch rate (the rate of wrong matching in the controllable relevance big data of foreign trade goods sales volume) [22]. In order to optimally describe the error relation, ω0 linear parameters (b1, b2, …, bn) are added to the mean square of the error. Then, the equations of reconfiguration error, feature point error and mismatch rate are shown in Eqs (16) ~ (18) respectively. They are CPW (v, u), APW (v, u) and WPR (v, u), specifically:

$$CPW(v,\;u)=\frac{M{\left(S_{i},\;S_{j}\right)}^{\lambda }\cdot \sqrt{CV(S_{i},\;S_{j})\omega_{0}+TCX{\left(S_{i}\right)}^{2}}}{CVV{\left(S_{i},\;S_{j}\right)}^{T_{i}}⊗TCZ(S_{i})\cdot TCL{(S}_{i}))}$$ (16)

$$APW(v,\;u)=\frac{\prod_{i=1}^{n}\;TCX{\left(Si\right)}^{3}\cdot M{\left(S_{i},\;S_{j}\right)}^{\omega_{0}/2}\cdot CPW(v,\;u)}{DT^{T_{i}}\cdot TCZ{\left(S_{i}\right)}^{\lambda /3}\cdot TCL(S_{i})}$$ (17)

$$WPR(v,u)=\frac{\sqrt[{T_{i}}]{TCL{\left(S_{i}\right)}^{3}\cdot TCX(S_{i})}}{APW(v,u)\cdot D{\mathrm{TT}}^{w_{0}}\cdot TCZ{\left(S_{i}\right)}^{b_{n}/4}}$$ (18)

Experiment 2 takes experiment 1 as the premise, and uses the above 10000 relevant data to do 10000 experiments again. The average value obtained is the final data. The performance of the DPMES and C&M-CVPDSS model is compared.

The indexes for evaluating the results of this experiment are as follows. Credibility measure is to describe the credibility of prediction results, and the reference value is 16 ~ 22; uncertainty discrimination [23] is the degree to distinguish other states of the prediction results, and the reference value is 10 ~ 15; the optimal search time is to measure the overall consumption of dynamic prediction, and the reference value is 10 ~ 15s; the error coefficient can be obtained by combining the equations of reconfiguration error, feature point error and mismatch rate [24], and the reference value is 5 ~ 7; controllable relevance degree is related to the above four indexes, and the reference value is 10 ~ 14. Eqs (19) ~ (23) are their equations respectively.


$$KXX(x)=\frac{TCZ(S_{i})\cdot \sqrt{TCL(S_{i})\cdot M{\left(S_{i},\;S_{j}\right)}^{\lambda }}}{{\left(CPW{\left(v,\;u\right)}^{\omega 0}+TCX{\left(S_{i}\right)}^{2}\right)}^{T_{i}}}$$ (19)

$$NQQ(x)=\frac{TCZ{\left(S_{i}\right)}^{T_{i}}\times TCL(S_{i})⊕M{\left(S_{i},\;S_{j}\right)}^{\lambda }}{APW{\left(v,\;u\right)}^{\omega 0}⊗TCX{\left(S_{i}\right)}^{b_{n}}}$$ (20)

$$ZJS(x)=\frac{TCZ(S_{i})bn\cdot TCL(S_{i})\omega 0}{WPR{\left(v,\;u\right)}^{T_{i}}\cdot \int_{0}^{b_{n}}KXX(x)}$$ (21)

$$WCXS(x)=\frac{APW(v,\;u)\cdot TCZ{\left(S_{i}\right)}^{\omega }\cdot NQQ{\left(x\right)}^{b_{n}}}{WPR(v,\;u)\cdot CPW(v,\;u)T_{i}\cdot \prod_{x=1}^{n}KXX(x)}$$ (22)

$$KKD(x)=\frac{WCXS(x)\cdot WPR(v,\;u)\cdot APW(v,\;u)}{NQQ{\left(x\right)}^{b_{n}}\cdot \sum_{x=1}^{n}\left(KXX(x)\cdot ZJS(x))\cdot CPW(v,\;u\right)}$$ (23)

In experiment 3, the future prediction efficiency of DPMES is investigated through outside sample prediction and fluctuation prediction of three platforms of C&M-CVPDSS model, cargo identification effectiveness prediction model, and DPMES.

Among them, the mean square error of prediction outside the fixed index sample is:

$$MSE(S_{i})=\frac{KXX(x)\cdot WCXS(x)\cdot TCL{\left(S_{i}\right)}^{T_{i}\cdot e}}{KKD(x)\cdot TCZ{\left(S_{i}\right)}^{\lambda }\cdot MAE}$$ (24)

Besides, the efficiency of parallel comprehensive volatility prediction is based on the actual dynamic sample information fixed in the platform and outside the platform in the early stage. Eqs (13) ~ (24) are adopted to predict the fluctuation of the prediction time period, and comprehensively test the prediction efficiency of the DPMES prediction effect on the fluctuation of export goods sales in the next year in parallel. The evaluation indexes include prediction error ratio (error ratio of overall prediction results), confidence (expressed as the confidence of prediction accuracy of recent export goods sales fluctuation), inventory optimization efficiency (inventory optimization cost performance according to comprehensive prediction results). Eqs (25) ~ (27) are related expression [25]:

$$YWP(x)=\frac{WCXS(x)⊕CPW{\left(v,\;u\right)}^{\lambda \cdot e}\cdot APW{\left(v,\;u\right)}^{T_{i}}}{TCZ{\left(S_{i}\right)}^{\lambda \cdot T_{i}}\cdot WPR(v,\;u)\cdot MSE(S_{i})}$$ (25)

$$ZXCD(x)=\frac{KXX(x)/CPW{\left(v,\;u\right)}^{\lambda \cdot T_{i}}\cdot APW{\left(v,\;u\right)}^{T_{i}}}{TCZ(S_{i})⊗NQQ{\left(x\right)}^{\lambda \cdot e}\cdot YWR(x)}$$ (26)

$$KCYR(x)=\frac{YWR(x)\cdot \sum_{i=1}^{n}TCX(S_{i})\cdot TCL{\left(S_{i}\right)}^{\lambda \omega })}{APW{\left(v,\;u\right)}^{T_{i}}\cdot TCZ(S_{i})\times ZXCD{\left(x\right)}^{\lambda \cdot e}}$$ (27)

## Results

### Experiment 1

Based on Figs 1 to 5, the dynamic prediction system is established by using java language in the front end and open source PHP and SQL Server in the background.

Fig 8 is an analysis of the test results. It shows that the reconfiguration error scatter diagram, feature point error scatter diagram and mismatch rate scatter diagram are all monotonic and parallel increasing forms. It can be said that the personalized prediction mechanism is closer to the actual prediction results when the scatter diagram is smoothly approaching; when the prediction efficiency of the previous normalized fitting data index on the fluctuation of export goods sales volume is analyzed, the prediction efficiency of the guidance method using the improved algorithm is the best. Hence, it can be said that the design of improved methods, personalized prediction mechanisms and intelligent prediction algorithms based on this premise is better.

**Fig 8:** Verification results of the improved algorithm.

### Experiment 2

Fig 9 is the experimental result of Experiment 2.

**Fig 9:** Performance comparison of various models (A: C&M-CVPDSS model; B: Prediction model of the actual effect of goods identification; C: DPMES).

Fig 9 reveals that when the fixed sales volume index is higher than the expected value and the goods sales tend to be hot, the prediction of incremental data is closer to the trend and accurate actual prediction value; on the contrary, the year-on-year reduction rate of sales will swing around the risk line. It suggests that the expected forecast of goods sales volume refers to the actual forecast index. The comprehensive prediction effect of DPMES is obviously better than the previous related models.

### Experiment 3

According to MSE (Si), the proportion of distributed quantitative and centralized qualitative errors in outside sample prediction is obtained. The following methods are adopted to compare the prediction results. The multidimensional decomposition method and connectability level of CV (Si, Sj) consider the interference of CVV (Si, SJ) on the error relationship. The prediction error of the next cycle reaches the highest when the year-on-year growth rate is low. Considering the interference of TCZ (Si) on the random prediction trust relationship, the prediction error has the ability of comparison. Figs 10 to 11 are prediction results.

**Fig 10:** DPMES prediction value based on sample data inside and outside the platform.

**Fig 11:** Confidence and inventory optimization efficiency of DPMES prediction results based on sample data inside and outside the platform.

Figs 10 and 11 reveal that the sale predication value of four quarters shows an upward trend; confidence and inventory optimization efficiency are generally acceptable values; besides, the predication error ratios from the first quarter to the fourth quarter are 2.3%, 2.1%, 2.4% and 2.4%, respectively, which are also in the acceptable range. On the premise of parallel prediction of each quarter, the cumulative growth rate of four quarters can be obtained by synthesizing the prediction results, which is very close to the actual results. Therefore, the DPMES prediction results based on the sample data inside and outside the platform have a better prediction accuracy for the fluctuation of sales volume of foreign trade goods. Based on the data of three experiments, the prediction accuracy and prediction efficiency of DPMES are highly improved, which can provide more reliable algorithm support for international trade.

## Conclusion

Under the background of world economic globalization, international trade is of great significance for a country to increase its foreign exchange reserves and enhance the market space and market competitiveness of its enterprises. In order to ensure the stable and rapid development of international trade and finance, it is particularly important to predict the sales trend of foreign trade goods in advance through the network model of the computer trade platform. Through the confidence of DPMES prediction results, inventory optimization efficiency and performance comparison experiments with other models, it is found that the performance of the designed model is better than that of other models. Thus, under the background of "Internet plus foreign trade" driving, the dynamic, intelligent, quantitative and qualitative prediction of foreign trade goods sales based on controllable relevance big data of foreign trade is realized. This has a certain reference value for foreign trade enterprises to make efficient marketing, formulate reasonable storage planning and reasonable financing of funds. However, since "Internet plus" and big data are all high-end computer technologies with relatively high difficulty, the design is only the initial application stage of "Internet plus" and big data technology. It is still difficult to realize the relevant innovations made in these computer science and technology in the design process, so it exerts an impact on the performance of the system. More in-depth study and discussion about the Internet plus foreign trade, big data technology and fusion algorithm will be conducted.

## Supporting information

S1 File (ZIP)
